# Characterization of air-liquid interface culture of A549 alveolar epithelial cells

**DOI:** 10.1590/1414-431X20176950

**Published:** 2017-12-11

**Authors:** J. Wu, Y. Wang, G. Liu, Y. Jia, J. Yang, J. Shi, J. Dong, J. Wei, X. Liu

**Affiliations:** 1 College of Clinical Medicine, Ningxia Medical University, Yinchuan, Ningxia, China; 2 Institute of Human Stem Cell Research, General Hospital of Ningxia Medical University, Yinchuan, Ningxia, China; 3 Center of Laboratory Medicine, General Hospital of Ningxia Medical University, Yinchuan, Ningxia, China; 4 Department of Pathology, Ningxia Medical University, Yinchuan, Ningxia, China; 5 College of Life Science, Ningxia University, Yinchuan, Ningxia, China

**Keywords:** Alveolar epithelium, A549 cells, Air-liquid interface, Alveolar epithelial type II cells, Alveolar epithelial type I cells

## Abstract

Alveolar epithelia play an essential role in maintaining the integrity and homeostasis of lungs, in which alveolar epithelial type II cells (AECII) are a cell type with stem cell potential for epithelial injury repair and regeneration. However, mechanisms behind the physiological and pathological roles of alveolar epithelia in human lungs remain largely unknown, partially owing to the difficulty of isolation and culture of primary human AECII cells. In the present study, we aimed to characterize alveolar epithelia generated from A549 lung adenocarcinoma cells that were cultured in an air-liquid interface (ALI) state. Morphological analysis demonstrated that A549 cells could reconstitute epithelial layers in ALI cultures as evaluated by histochemistry staining and electronic microscopy. Immunofluorescent staining further revealed an expression of alveolar epithelial type I cell (AECI) markers aquaporin-5 protein (AQP-5), and AECII cell marker surfactant protein C (SPC) in subpopulations of ALI cultured cells. Importantly, molecular analysis further revealed the expression of AQP-5, SPC, thyroid transcription factor-1, zonula occludens-1 and Mucin 5B in A549 ALI cultures as determined by both immunoblotting and quantitative RT-PCR assay. These results suggest that the ALI culture of A549 cells can partially mimic the property of alveolar epithelia, which may be a feasible and alternative model for investigating roles and mechanisms of alveolar epithelia *in vitro.*

## Introduction

Alveoli are the main terminal structures of distal airway for gas exchange and the units of lung function. The surfaces of alveoli are composed of two types of epithelial cell: alveolar type I cells (AECI) and alveolar type II (AECII) cells (1). AECI cells are applanate-shaped cells and cover 95% of the alveolar surface of the lung, although they are in fewer number than AECII cells. The major function of AECI cells is gas exchange, and ion and fluid balance maintenance (2). AECII cells, however, are large and cuboidal-shaped cells, and cover a much smaller percentage of alveolar surfaces. Of note, AECII cells are specialized epithelial cells for maintaining lung function and homeostasis. AECII cells can secrete active substance and regulate the metabolism of alveolar surfactant, express innate immune molecules, and regenerate and restore alveoli in response to an injury. Importantly, a subset of AECII cells has been characterized as epithelial progenitors or stem cells with a capacity to differentiate into AECI cells or give rise to new AECII cells during alveolar injury repairs (3,4).

Indeed, AECII cells are one of the most investigated cell types for understanding the physiological and pathological mechanisms of many pulmonary diseases, such as lung cancer and pulmonary fibrosis. To this end, a method for the isolation and culture of AECII cells mimicking alveolar microenvironment *in vivo* is becoming essential. However, this technology has not been implemented yet, partially owing to primary AECII cells losing their phenotype and expression of cell markers during the traditionally submerged culturing *in vitro* (5). In addition, alternative strategies using immortalized or tumor AECII cell lines also fail to fully differentiate into alveolar epithelial cell phenotypes that are seen *in vivo* (5). Therefore, culturing alveolar epithelial cells in submerged cell-culture conditions is an ineffective and artificial environment (6). To better mimic the *in vivo* environment of alveolar epithelial cells, *in vitro* models including 3-dimensional cultures under airflow, air-liquid interface culture, with tissue stretching and movement have been developed (4).

However, a compelling body of studies have successfully demonstrated the isolation and *in vitro* culturing of AECII cells for many species, including human, mouse, pig, and rat. Moreover, the air-liquid interface (ALI) cultures using rat and human AECII cells demonstrated the potential of AECII cells to differentiate into AECI cells *in vitro* (7). However, unlike the feasibility and availability of isolating and ALI-culturing human primary epithelial cells from large airway, such as tracheal, bronchi and bronchioles (8), the isolation and long-term culturing to obtain sufficient AECII for ALI culturing are difficulty and currently infeasible. Therefore, submerged cultures of immortalized or tumor AECII cell lines, such as A549 cells are currently used as models of alveolar epithelia in most *in vitro* studies. The objective of this study was to characterize the epithelial property of A549 cells cultured under an ALI condition.

## Material and Methods

### Cell culture

Human adenocarcinoma A549 (ATCC# CCL-185) cell line was purchased from American Type Culture Collection (ATCC, USA). Cells were cultured in 1640 medium (Gibco, USA) supplemented with 10% fetal bovine serum (FBS) and 1% penicillin-streptomycin and maintained at 37°C incubator in atmosphere of 5% CO_2_. For generation of ALI cultures, membranes of Millicell inserts (0.4-mm pore, polycarbonate, Millipore, USA) were pre-coated with 70 µg/mL of type I rat tail collagen (BD Biosciences, USA), single cell suspension of A549 cells were seeded on apical surfaces of collagen-pre-coated membranes with densities of 3×106 and 0.5×106 cells per well for diameters of 30 and 12 mm inserts, respectively. The culture medium of the apical side was removed at 24 h after the seeding to establish an ALI condition. The ALI cultured cells were refreshed with medium in the bottom of insert at two-day intervals (9,10).

### Hematoxylin and eosin histochemical staining

After 2-weeks culturing, ALI culture inserts were fixed with 4% paraformaldehyde, and dehydrated in gradient alcohol series before they were embedded in paraffin. Sections of 4-μm thickness were employed for hematoxylin and eosin (HE) staining. The morphology of cells was observed under the Olympus BX43 light microscopy equipped with DP-73 camera (Olympus China, Shanghai, China).

### Immunofluorescence staining

Immunofluorescent staining was applied to determine the expression of AECII cell marker surfactant protein C (SPC) and AECI cell marker aquaporin-5 (AQP-5). The membranes of 2-week ALI cultures were fixed in filtered 4% paraformaldehyde at room temperature for 15 min prior to be washed for 3×3 min with PBS. The cells were then permeabilized with 0.2% Triton X-100 for 20 min at room temperature, followed by blocking with 5% normal donkey serum in PBS at room temperature for 60 min, after which they were incubated with primary antibodies against SPC (1:1000, Merck Millipore, USA) or AQP-5 (1:500, Abcam, USA) in PBS at 4°C overnight. Following extensive washing for 3×10 min with PBS to remove primary antibodies, the membranes were incubated with Alexa Fluor 488-labelled donkey-anti-rabbit IgG secondary antibody (1:500, Jackson ImmunoResearch Laboratories, USA) at room temperature for 60 min. The stained membranes were then mounted on slides with Vectashield Mounting Medium containing DAPI (Vector Laboratories, USA), and covered with a coverslip after washing in PBS for 3×5 min. Images were acquired by Leica TCS SP2 A0BS Confocal System and processed on Leica Confocal Software v.2.6.1 (Leica, Germany).

### Electron microscopy

Scan electron microscopy (SEM) and transmission electronic microscopy (TEM) were employed for morphological evaluation of cell differentiation after 2 weeks post-seeding. For SEM, 2-week-old ALI culture inserts were rinsed twice in PBS and fixed in 3.5% glutaraldehyde in 0.15 M phosphate buffer, pH 7.4, at room temperature for 1 h. They were then dehydrated in gradient ethanol series and treated with hexamethyldisilazane. After air-dried at room temperature, the membrane was sputter-coated with platinum/palladium prior to be visualized on a Hitachi S-3400 Microscope (Hitachi LTD, Japan) (11). For TEM, the membranes were first fixed as for SEM, followed by infiltration with Spurr resin following dehydration. Serial sections of 80 nm were then viewed on a Hitachi H-7000 Electron Microscope (Hitachi LTD) (12,13).

### Immunoblotting analysis

Whole cell extracts were prepared homogenizing cells in RIPA buffer for 3.5 h on ice. The cell lysate was centrifuged at 12,000 *g* for 30 min at 4°C for clarifying. The resultant supernatant of lysates (45 µg) were resolved on 10% sodium dodecyl sulfate polyacrylamide gel (SDS-PAGE) and transferred to PVDF membranes (Millipore). The membranes were blocked with 5% fat-free dry milk in PBS containing 0.1% Tween-20 for 1 h at room temperature, and probed with primary antibodies to proteins of interest at 4°C overnight. Then the membranes were incubated with appropriate horseradish peroxidase labeled secondary antibodies for 1 h at room temperature. The blots were then developed using the enhanced Western Bright ECL reagent (Advansta Inc., USA). The levels of protein expression were semi-quantified by absorbance using ImageJ Software version 1.46 (http://rsb.info.nih.gov/ij/). The ratio between the net intensity of each sample divided by the β-actin internal control was calculated as densitometric arbitrary units (AU) which served as an index of relative expression of a protein of interest (14,15). The primary antibodies used in this study were rabbit anti-SP-C (1:1000, Merck Millipore, USA), rabbit anti-AQP-5 (1:1000, Abcam, USA), mouse anti-thyroid transcription factor-1 (TTF-1; 1:1000, Thermo Fisher Scientific, UK), rabbit anti-zonula occludens-1 (ZO-1; 1:1000, Zymed Lab Inc., USA), rabbit anti-Mucin 5B (MUC5B; 1:1000, Santa Cruz Biotech, USA) and rabbit anti-β-actin (1:1000, Santa Cruz Biotech).

### RNA isolation and real-time quantitative RT-PCR

The total RNA from differently treated cells was purified using Trizol reagent per manufacturer's instruction (Invitrogen, USA). The quality of RNA was assayed by calculation of the RNA integrity number (RIN). High quality RNA (RIN value greater than 9.0) was used for reverse transcription of first-strand cDNA synthesis by reverse transcription using M-MLV reverse transcriptase (TransGen Biotech, China), and the transcript expression of the gene of interest was amplified using TransStart Tip Green qPCR SuperMix (TransGen Biotech) in LightCycler 480 II PCR system (Roche Diagnostics, Switzerland). The thermal cycling condition for PCR amplification was 95°C for 30 s, 40 cycles of 95°C for 5 s, 60°C for 20 s, and 72°C for 20 s, followed by 40°C for 20 min. The primer sets used for RT-PCR were designed and synthesized in Shanghai Sangon Biotech Inc. (China) by bioinformatics tools using available mRNA sequences. The sequences of primers are listed in Table 1. The internal controls were always included to normalize each reaction with respect to RNA integrity, sample loading and inter-PCR variations. The relative expression ratio was calculated from the real-time PCR efficiencies and the crossing point deviation of a given gene *vs*. β-actin. In each independent experiment, the mean gene expression ratios obtained with regular submerged cultures were given a value of 1 (fold). The specificity of PCR was determined by sequencing of the PCR products.

**Table 1.** Sequences of primer sets used in this study.

Gene	Forward primer (5′-3′)	Reverse primer (5′-3′)
SP-C	CCTGAAACGCCTTCTTATCG	CTCCAGAACCTACTCCGTGT
AQP-5	ATGGTGGTGGAGCTGATTCT	GGTGACAGACAGGCCAATG
ZO-1	ATGACTCCTGACGGTTGGTC	CACAGTTTGCTCCAACGAGA
MUC5B	CCACAGCTACCAGCGTTACA	TGGAGTAGAGGAGGGTGTGG
TTF-1	GGCATTGAGAGTGCAGACAA	GGGCAATGTTCCCACCAATG
β-actin	CTCTTCCAGCCTTCCTTCCT	AGCACTGTGTTGGCGTACAG

### Statistical analysis

All data collected in this study was obtained from at least three independent experiments for each condition. SPSS19.0 analysis software (USA) and PRISM 5 (Graphpad, USA) were used for the statistical analysis. Statistical evaluation of the data was performed by one-way ANOVA when more than two groups were compared with a single control, and *t*-test was employed for comparison of differences between two groups. P<0.05 was considered as a statistically significant difference. Data are reported as means±SD.

## Results

### Morphological analysis of A549 cell ALI cultures

In order to characterize ALI culture of A549 cells, A549 cells were seeded on collagen-pre-coated membranes of Millicell inserts and cultured in an air-liquid interface phase. The cells were evaluated for alveolar epithelial cell phenotypes by ascertaining their morphology and the expression of cell type-specific markers at different time points using appropriate assays (Figure 1A). Morphological analysis revealed the formation of an intact epithelial cell layer on the membrane as seen by HE staining (Figure 1B). The conventionally submerged culture cells exhibited inerratic shapes with smooth surface, but ALI cultured cells displayed anomalous shapes and rough cell surfaces with abundant secretions observed under a scanning electron microscopy (Figure 2). Morphological analysis using transmission electron microscopy further revealed that the submerged cell cultures exhibited clear border and organelles, and were lacking obvious microvilli, although they had AECI-like outward appearance in some extent (16) (Figure 3A, C and E). However, the ALI cultured cells were more compacted with clear cell junctions and abundant mucus on the apical surface (Figure 3B, D and F).

**Figure 1.** The experimental process and histochemical staining. *A*, Experimental design and process. A549 cells were seeded on collagen pre-coated membranes of Millicell inserts, and cultured under an air-liquid interface (ALI) state for the indicated times. Membranes were then collected for morphological and molecular analysis. *B*, Morphological evaluation of a 2-week-old A549 epithelial cell ALI culture by hematoxylin and eosin staining, showing the epithelial layer of A549 cells grown on the membranes.

**Figure 2.** Scanning electronic microscopy (SEM) of air-liquid interface (ALI) of 2-week-old A549 ALI cultures and logarithmic phase of submerged cultures. *A*, *C*, and *E*, Different magnifications of submerged cultures showing a morphology of inerratic shapes with smooth surfaces; *B*, *D*, and *F*, different magnifications of ALI cultures exhibiting anomalous shapes and rough cell surfaces with abundant secretion on the surface of culture. Magnification: A and B=50 μm; C and D=10 μm; E and F=5.0 μm.

**Figure 3.** Transmission electron microscopy (TEM) of air-liquid interface (ALI) cultures and logarithmic phase of submerged cultures of A549 cells. *A*, *C*, and *E*, Different magnifications of submerged cultures showing a morphology of clear border and organelles and lack of obvious microvilli, although they had AECI-like outward appearance in some extent; *B*, *D*, and *F*, different magnifications of ALI cultured cells displaying a more compacted morphology with clear cell junction and abundant mucus on the apical surface. Magnification bars: A and B=5000 nm; C and D=2000 nm; E and F=1000 nm.

### Immunological characterization of A549 cell ALI cultures

To further characterize A549 cells in ALI cultures, immunofluorescent staining assay was used to determine the expression of cell-specific markers of AECI and AECII cells. As expected, the expression of AECI cell specific marker AQP-5 and AECII cell marker SP-C were observed on the cytomembrane and in the cytoplasm of subset cells, respectively (Figure 4).

**Figure 4.** Expression of alveolar epithelial cell type markers determined by immunofluorescent staining. Two-week-old membranes of A549 air-liquid interface (ALI) cultures were used for determination of the expression of AECI cell specific marker aquaporin-5 (AQP-5) and AECII cell marker surfactant protein C (SP-C) by immunofluorescent staining assay. The expression of both of AQP-5 and SPC was observed on the cytomembrane and in the cytoplasm of distinct subset cells, respectively. Magnification bars: 25 µm.

### Molecular characterization of A549 cell ALI cultures

AECII cells were reported to lose phenotype markers over time when they were cultured in monolayer (17), but they might be able to express cell type-specific markers in an ALI interface culture (4). Therefore, we sought to analyze the expression of epithelial cell markers in both transcriptional and translational levels by qRT-PCR and immunoblotting assays, respectively. Indeed, transcriptional analysis revealed that significantly more transcripts of SPC, AQP-5, TTF-1, MUC5B and ZO-1 were detected in ALI cultures compared to submerged cultures, particularly in the 2-week-old ALI cultures (Figure 5). However, a dynamic change in proteins of epithelial markers was observed in A549 cell ALI cultures as determined by the immunoblotting assay. The overall SPC protein was moderately increased in ALI cultures in comparison with submerged cultures. Consistently, the AECI cell marker proteins AQP5 and TTF-1 were also increased in ALI cultures compared to submerged cultures. An increased mucin 5B (MUC5B) was also observed in ALI cultures. Interestingly, the epithelial tight junction protein ZO-1 was detected in both ALI cultures and submerged cultures, except it failed to be detected in ALI cultures of 3 days. All the above examined proteins of interest were found increased in ALI cultures of 1 and 2 weeks, compared with submerged cell cultures (Figure 6), suggesting that 1-2 weeks was the best window for the alveolar property of the A549 ALI culture model. Together with the aforementioned morphological data, this result suggested that A549 cells might partially maintain alveolar epithelial cell properties in ALI state.

**Figure 5.** Transcripts of several key genes of interest in A549 cell air-liquid interface (ALI) cultures at 3 days, 1 week, 2 weeks, and 3 weeks were examined by a qRT-PCR assay. A significantly induced expression of SP-C (*A*), AQP-5 (*B*), TTF-1 (*C*), and ZO-1 (*D*) mRNAs were observed in ALI cultures compared to submerged cultures of A549 cells (control, C), particularly in the 2-week-old cultures. Data are reported as means±SD from 3 independent experiments (n=9)., D: days; W: week(s). *P<0.05 and **P<0.01 compared to the submerged culture control (ANOVA).

**Figure 6.** Protein of several key cell-specific markers of alveolar epithelial cells in A549 cell air-liquid interface (ALI) cultures at 3 days, 1 week, 2 weeks and 3 weeks were examined by an immunoblotting assay using specific antibodies. *A*, Representative blots of immunoblotting assay showing significantly higher levels of AECI cell type markers AQP-5, TTF-1, and epithelial cell proteins MUC5B and ZO-1 observed in ALI cultures compared to submerged cultures of A549 cells (control, C). However, AECII cell type-specific marker SPC was only moderately increased in ALI cultures compared to submerged cultures of A549 cells. *B*, Densitometry values are reported as fold-change for SPC, AQP-5, TTF-1, MUC5B and ZO-1 proteins over β-actin. Data in *B* are reported as means±SD from 3 independent experiments (n=3). D: days; W: week(s). *P<0.05 and **P<0.01 compared to the submerged culture control (ANOVA).

## Discussion

The purpose of this study was to characterize alveolar epithelial properties of a three-dimensional (3D) ALI culture of A549 cells. Subpopulations of ALI cultured A549 cells exhibited abilities to partially express cell type-specific markers of AECI and AECII cells. The ALI culture model has several advantages compared to submerged cultures of immortalized or tumor cell lines. Therefore, ALI epithelial culture of A549 cells might be a potentially useful and feasible *in vitro* model for investigating the physiological and pathological roles of alveolar epithelial cells in human lungs. In addition, the ALI culture of A549 cells would better mimic alveolar epithelia compared to the submerged A549 cell cultures.

AECII cells have a potency to give rise to new AECII cells and differentiate into AECI cells during alveolar injury repair and regeneration, therefore they have been considered progenitor cells in the alveoli (3,4,18). Previous studies have demonstrated that primary AECII cultured under a conventional or submerged cell culture condition showed a loss of AECII cell phenotype and of the surfactant synthesis capacity, and cell morphology alteration (19). A compelling body of studies has demonstrated the capacity of primary airway epithelial cells to reconstitute airway epithelia of many species in ALI culture models, including human (10), sheep (11), bovine (14), mouse (13), non-human primate (20), pig and ferret (9). Primary airway epithelial cells isolated from large airways, such as the trachea and bronchus of different species, are able to fully differentiate into various epithelial cell types in ALI culture model, which is considered an organotypic model (21). Despite AECII cells isolated from bovine (22), human (1,23,24), pig (25,26), mouse (27), and rat (7) lungs exhibited the ability to maintain their cell phenotype in an ALI culture model (7,24), it remains a great challenge to isolate or culture sufficient AECII cells for generation of ALI cultures. Therefore, there is a need to develop an alternative model for investigating roles and mechanisms of alveolar epithelia. In the present study, the characterization of A549 cells cultured in an ALI phase was examined. The results showed that the expression of alveolar epithelial type I cell markers AQP-5 and TTF-1 was significantly increased in ALI cultures as compared with submerged cultured A549 cells. In addition, mucin 5B and ZO-1 were determined in the ALI cultures, but the expression of AECII cell marker SPC was only moderately increased.

A previous study has suggested that dipalmitoyl phosphatidyl choline-containing multilamellar bodies (MLB) are ultrastructural hallmark of AECII cells (28). The other hallmark of AECII cells includes lipids, which are major components of pulmonary surfactant that are able to prevent alveoli from collapse by reducing alveolar surface tension at the end of expiration (28). In addition, lysosomes have also been thought as an origin of MLB, and a long-term culture of A549 cells may lead the accumulation of lysosomes (28). In agreement with these findings, the morphological analysis of electron microscopy also revealed a large number of lipid droplets and lysosomes in the cytoplasm in the 2-week-old ALI culture of A549 cells (28). Equally noteworthy, A549 cells are adenocarcinoma cells with unlimited capacity of proliferation, but limited differentiation, although they have been widely used as an AECII cell models *in vitro* (29). In line with this, we also noted that a higher level of alveolar epithelial cell markers was determined in 1- to 2-week-old ALI cultures of A549 cells rather than cultures of an earlier or later time period. We reasoned that A549 cells could differentiate into alveolar epithelial cell types at some extent in early time points, but they might retain their carcinoma cell properties along with a reduced capacity of differentiation in a long-term ALI culture. However, the exact mechanism of this phenotype of cultures need to be further investigated. The 1- to 2-week window for the best alveolar properties of A549 ALI culture model limits the use of this model in studies that a long-term follow up is required. In addition, despite an increased expression of AECI cell type markers AQP-5 and TTF-1 being observed in ALI-cultured A549 cells, AECI cells have not been morphologically identified. This also implies a limitation of ALI cultures generated from A549 cells and a necessity of primary AECII cells for generation of alveolar epithelial model *in vitro*.

Collectively, in the present report, an ALI epithelial culture model of A549 cells was characterized. The results revealed an induced expression of alveolar epithelial specific cell markers AQP-5 and SPC in ALI cultured A549 cells, indicating partial alveolar epithelial cell properties. These results thus suggest that the ALI-cultured A549 cells may be a feasible and alternative model for investigating roles and mechanisms of alveolar epithelia *in vitro.*
